The article "Electroacupuncture Ameliorates Depression-Like Behaviour in Rats by Enhancing Synaptic Plasticity via the GluN2B/CaMKII/CREB Signalling Pathway" was published in 2021. Journal: Evid Based Complement Alternat Med.

# Electroacupuncture Ameliorates Depression-Like Behaviour in Rats by Enhancing Synaptic Plasticity via the GluN2B/CaMKII/CREB Signalling Pathway

**DOI:** 10.1155/2021/2146001

**Published:** 2021-11-03

**Authors:** Kun Zhang, Ran Liu, Jingruo Zhang, Xifang Wei, Yuan Gao, Wen Ma, Yijing Li, Wa Cai, Weidong Shen

**Affiliations:** ^1^Department of Acupuncture, Shuguang Hospital affiliated to Shanghai University of Traditional Chinese Medicine, Shanghai, China; ^2^Institute of Acupuncture and Anesthesia, Shuguang Hospital affiliated to Shanghai University of Traditional Chinese Medicine, Shanghai, China

## Abstract

**Background:**

Hippocampal synaptic plasticity during the pathological process of depression has received increasing attention. Hippocampal neuron atrophy and the reduction in synaptic density induced by chronic stress are important pathological mechanisms of depression. Electroacupuncture (EA) exerts beneficial effects on depression, but the mechanism is unclear. This study explored the effect of EA on synaptic plasticity and the potential mechanism.

**Methods:**

Forty-eight SD rats were randomly divided into the control, chronic unpredictable mild stress (CUMS), EA, and fluoxetine (FLX) groups, and each group consisted of 12 rats. The sucrose preference test, open field test, and forced swimming test were used for the evaluation of depression-like behaviour, and Golgi and Nissl staining were used for the assessment of synaptic plasticity. Western blotting and immunofluorescence were conducted to detect proteins related to synaptic plasticity and to determine their effects on signalling pathways.

**Results:**

We found that CUMS led to depression-like behaviours, including a reduced preference for sucrose, a prolonged immobility time, and reduced exploration activity. The dendritic spine densities and neuron numbers and the protein levels of MAP-2, PSD-95, and SYN were decreased in the hippocampi of rats with CUMS-induced depression, and these trends were reversed by EA. The molecular mechanism regulating this plasticity may involve the GluN2B/CaMKII/CREB signalling pathway.

**Conclusion:**

These results suggest that EA can improve depression-like behaviour and hippocampal plasticity induced by CUMS, and the mechanism may be related to the GluN2B/CaMKII/CREB pathway.

## 1. Introduction

Depression is a common serious mental disease that mainly manifests as a depressed mood, declining interests, a lack of pleasure, serious insomnia, stupor and other somatic symptoms, and even suicide [1, 2]. The depression prevalence rate continues to increase, and the disease poses substantial social and economic burdens. According to World Health Organization statistics, depression accounts for nearly 4.3% of the global disease burden and is expected to rank first in 2030 [3, 4]. At present, the commonly used antidepressants in the clinic have some limitations, such as delayed responses and low effective rates [5–7], and are often accompanied by some side effects, such as gastrointestinal reactions, palpitations, and drowsiness [8–10]. Considering the increasing incidence rate of depression and the challenges of traditional antidepressants, more effective treatments are urgently needed.

The exact mechanisms of depression pathogenesis remain to be identified. In recent years, hippocampal synaptic plasticity has received more attention with respect to the pathological process of depression [11, 12]. Numerous studies have confirmed that depression is directly related to the abnormal regulation of synaptic plasticity. Imaging studies have shown that the hippocampal volume of patients with depression is significantly lower than that of healthy subjects [13]. Studies have found that acute and chronic stress can cause the shrinkage and loss of hippocampal neurons and glial cells, which results in neuronal atrophy and decreased synaptic density [14–16]. The levels of various proteins that serve as markers of synaptic plasticity, such as microtubule-associated protein 2 (MAP-2), postsynaptic density 95 (PSD-95), and synaptophysin (SYN), are decreased in the hippocampus [17], and the severity of depression is significantly related to the number of hippocampal spine synapses [18, 19]. Antidepressant therapy has also been found to work by regulating neuroplasticity [20, 21]. Based on these results, synaptic plasticity in the hippocampus is closely related to the occurrence of depression.

N-methyl-D-aspartic acid receptor (NMDAR) is an ionic glutamate receptor, and acute or chronic stress increases the levels of glutamate around synapses in the hippocampus and, thereby, leads to NMDAR overactivation [22, 23], which is an important factor in inducing depression. As a regulatory subunit, GluN2B plays an important role in regulating synaptic plasticity, learning, and memory [24, 25]. More importantly, a recent study reported that the expression of GluN2B is significantly upregulated in the hippocampus of rats with CUMS-induced depression, and specific inhibitors of GluN2B exhibit good antidepressant effects [26]. These studies suggest that GluN2B and its signalling pathway in synaptic plasticity may be a potential target in antidepressant research [27].

Acupuncture is a widely used supplementary and alternative strategy for the treatment of various mental and emotional disorders (including depression, anxiety disorders, posttraumatic stress disorder, and sleep disorders), and numerous clinical studies have shown that acupuncture has good effects on depression [28–30]. However, the mechanism of the antidepressant action of acupuncture remains poorly understood. We infer that the antidepressant effect of acupuncture is related to synaptic plasticity mediated by the GluN2B pathway. In this study, we established a model of chronic unpredictable mild stress (CUMS) depression to explore the effects of acupuncture on behaviour. Moreover, hippocampal synaptic plasticity and the downstream regulation of GluN2B were explored to clarify the mechanism of acupuncture in the treatment of depression.

## 2. Materials and Methods

### 2.1. Animals and Groups

Male Sprague Dawley rats weighing 180–200 g were raised at the Experimental Animal Center of Shanghai University of Traditional Chinese Medicine. The experiment was approved by the Animal Research Ethics Committee of Shanghai University of Traditional Chinese Medicine (PZSHUTCM200814011). All animals were housed under controlled temperature (23 ± 1°C) and light (12 h light/dark cycle) conditions and were adaptively fed for one week before the formal experiment. The experimental animals were randomly divided into 4 groups (12 rats in each group): the control, CUMS, EA, and fluoxetine (FLX) groups. The rats in the control group were fed normally without any intervention, and those in the CUMS, EA, and FLX groups were exposed to chronic unpredictable mild stress for 21 days and then subjected to behavioural tests. After successful modelling, the rats in the CUMS group were not administered any treatment, and those in the electroacupuncture group were subjected to electroacupuncture intervention for 21 days. The rats in the fluoxetine group were administered fluoxetine by gavage for 21 days (10 mg/kg/day). The experimental procedure is shown in Figure 1.

### 2.2. CUMS Procedure

The CUMS protocol was slightly modified according to a previous study [31, 32], and two stressors were randomly administered every day for 21 days. The stress programme included 24 h of fasting, 24 h of water deprivation, 24 h of cage tilting at 45°, soiled bedding/wet bedding, 24 h of a reversed light/dark cycle, 24 h of crowding, 4 min of cold swimming (4°C)/forced cold swimming (4°C), 2 h of physical restraint, 1 h of cold immobilization at 4°C, and 4 h of flashing.

### 2.3. Acupuncture Treatment

The rats were first fixed on a special fixator, and acupuncture needles (0.22 mm × 25 mm, Huan-Qiu, Suzhou Huanqiu Medical Appliance Co., Ltd., China) were inserted into the GV20 and GV29 acupoints (Figure 2) at depths of 7 mm and 4 mm and connected to an electroacupuncture apparatus (Hwato SDZ-V, Suzhou Medical Supplies, China). The parameters of the electroacupuncture apparatus were determined according to our previous research [33]. Specifically, the waveform was an intermittent wave, the frequency was 2 Hz, and each EA treatment lasted for 20 min.

### 2.4. Behaviour Tests

#### 2.4.1. Sucrose Preference Test

The sucrose preference test (SPT) was slightly modified as described above [26, 34]. First, all the rats were given 2 bottles of 1% sucrose solution for 24 h. The rats were then given 1 bottle of water and 1 bottle of 1% sucrose solution for 12 h, followed by changing the positions of the water and sucrose bottles for 12 h. The rats were subsequently deprived of water for 24 h and then given a bottle of 1% sucrose solution and a bottle of water for 2 h, and the consumption of sucrose solution and water was recorded.

#### 2.4.2. Open-Field Test

We evaluated the locomotor activity of the rats via the open-field test (OFT). The OFT apparatus consisted of a 100 cm × 100 cm × 50 cm plastic board, and the floor was divided into 25 equal squares. The rats were placed at the centre of the device and allowed to freely explore the platform for 5 min. The numbers of crossings and rearings were recorded using SuperMaze 2.0 (Shanghai Xin-ruan Information Technology Co., China). The number of times the rats passed through the bottom surface (three claws were all entered into the square) was counted as the number of crossings, and the number of times the rats assumed an erect posture (two front paws vacating or climbing the walls of box) was counted as the number of rearings. Before each test, the equipment was wiped clean to remove any residual odour.

#### 2.4.3. Forced Swim Test

The forced swim test (FST) was performed as previously reported [33]. The rats were placed in a bucket (height of 50 cm × diameter of 25 cm) with a water depth of 35 cm (20–22°C) and allowed to swim for 6 min. The immobility of each rats, which was defined as no movements other than those necessary to maintain its head above water, was recorded during the last 4 min. The immobility time was recorded by two observers who were blinded to the groupings.

### 2.5. Western Blot Analysis

Hippocampal tissue was cut into small pieces and homogenized with RIPA lysis buffer (P0013C, Beyotime, China). After centrifugation at 12000 rpm for 10 min, the supernatant was collected, and the protein concentration in the supernatant was determined using a BCA protein concentration assay kit (P0012S, Beyotime, China). Forty micrograms of protein was electrophoretically separated by SDS-PAGE and then transferred to PVDF membranes (Millipore, China). The membranes were blocked for 1 h at room temperature using 5% skim milk powder in PBS containing 0.1% Tween 20 (PBST). The following primary antibodies were used: anti-PSD-95 (GB11277, 1 : 1000, Servicebio Technology), anti-SYN (GB11553, 1 : 1000, Servicebio Technology), anti-MAP-2 (GB11128-2, 1 : 1000, Servicebio Technology), anti-GluN2B (ab28373, 1 : 1000, Abcam), anti-CaMKII (sc-376828, 1 : 1000, Santa Cruz Biotechnology), anti-p-CREB (ab32096, 1 : 1000, Abcam), anti-CREB (ab32515, 1 : 1000, Abcam), and anti-*β*-actin (66009-1-Ig, 1 : 5000, ProteinTech Group). The membranes were washed with PBST (10 min, 3 times) and then incubated with a horseradish peroxidase-conjugated secondary antibody for 1 h at room temperature. The blots were subsequently detected using an enhanced chemiluminescence kit and analysed with ImageJ software.

### 2.6. Immunofluorescence Staining

After the last behavioural tests, the rats were immediately anaesthetized via an intraperitoneal injection of 2% pentobarbital sodium followed by 50 ml of 0.9% normal saline and 150 ml of 4% paraformaldehyde. Their brain tissues were then rapidly removed, fixed with precooled paraformaldehyde for 48 h, dehydrated, embedded, and coronally sectioned. First, the paraffin sections were dewaxed with xylene (15 min, twice), an ethanol gradient (100%, 85%, and 75%, 5 min, once with each), and distilled water (5 min, once). The slides were then boiled in citric acid at pH 6 for 10 min for antigen repair, blocked with 3% BSA for 10 min, incubated overnight with a primary antibody (PSD-95, 1 : 200; SYN, 1 : 500; and MAP-2, 1 : 500; Servicebio, China) at 4°C, and washed with phosphate buffered saline (PBS) (5 min, 3 times). The secondary antibody of the corresponding species of the primary antibody was added, and the membranes were incubated at room temperature in the dark for 50 min, washed in PBS (5 min, 3 times), and incubated with DAPI, and the mean fluorescence intensity was quantified using ImageJ (version 1.51).

### 2.7. Nissl Staining

Paraffin sections were dewaxed with xylene (3 times, 10 min each time), an ethanol gradient (100%, 5 min; 90%, 2 min; 70%, 2 min) and distilled water (5 min). The tissue sections were stained with 0.5% toluidine blue (Servicebio Technology) at room temperature for 1 min, dehydrated with 95% ethanol, baked at 65°C for 4 h, cleared with xylene for 10 min, and sealed with neutral gum. Images of the hippocampal CA3 region were obtained under a light microscope (Nikon Eclipse E100), and the number of nerve cells was counted using ImageJ.

### 2.8. Golgi Staining

After the rats were sacrificed, their brain tissues were rapidly removed, fixed in 4% paraformaldehyde solution for 24 h, cut into sections with a thickness of 2-3 mm, and immersed in Golgi staining solution (Servicebio, China). The staining solution was replaced with fresh solution after 48 h and then every three days over a 14-day period. The tissue was removed, placed in 15% sucrose solution, dehydrated at 4°C in the dark for approximately 1 day, placed in 30% sucrose solution, and dehydrated at 4°C in the dark for 2 days. The tissue block was removed, washed with distilled water for 1 min, placed in 75% glacial acetic acid for 36 h, washed with distilled water for 1 min, cut into 100 *μ*m-thick sections with a vibration slicer (Leica vt1000s), and dried overnight. The slices were soaked in distilled water for 4 min, dipped in concentrated ammonia for 10 min, washed in distilled water for 4 min, and sealed with glycerin gelatine. Images were acquired with a light microscope (Nikon Eclipse E100), and the dendritic spine density was calculated by dividing the number of dendritic spines by their length.

### 2.9. Statistical Analysis

All experiments were statistically analysed using GraphPad Prism 9 software (San Diego, California, America). The experimental data are expressed as the means ± SEMs. Differences among multiple groups were determined by one-way ANOVA followed by Tukey's post hoc test if the F value indicated significance. *P* < 0.05 was considered to indicate statistical significance.

## 3. Results

### 3.1. EA Reversed CUMS-Induced Depression-Like Behaviours

The OFT results showed that the numbers of crossings and rearings showed significant differences among the groups after 21 days of CUMS exposure (F (3, 44) = 36.64, *P* < 0.0001; F (3, 44) = 17.63, *P* < 0.0001). Similarly, significant differences in the numbers of crossings and rearings were found among the groups on the 42nd day (F (3, 44) = 9.415, *P* < 0.0001; F (3, 44) = 9.472, *P* < 0.0001), and the EA and FLX groups exhibited significantly increased numbers of crossings and rearings compared with the model group (*P* < 0.05, *P* < 0.05, Figures 3(a) and 3(b)). The SPT results showed that the ratios of sucrose consumption were significantly different after 21 days of CUMS exposure (F (3, 44) = 13.15, *P* < 0.0001). On the 42nd day, a significant difference in the ratios of sucrose consumption was found among the groups (F (3, 44) = 16.06, *P* < 0.0001). The treatments with EA and FLX increased sucrose consumption compared with the CUMS group (*P* < 0.05, *P* < 0.05, Figure 3(c)). The FST results revealed that the immobility times the among groups were significantly different after 21 days of CUMS exposure (F (3, 44) = 15.10, *P* < 0.0001). On the 42nd day, a significant difference in the immobility time of the rats was found among the groups (F (3, 44) = 7.966, *P*=0.0002). The immobility time of the rats in the EA and FLX groups was significantly lower than that of the rats in the model group (*P* < 0.05, *P* < 0.05, Figure 3(d)).

### 3.2. EA Increased the Expression of Synaptic Plasticity-Related Proteins

We investigated the effects of EA on synaptic plasticity-related proteins. First, the effects of EA on the synaptic plasticity-related proteins MAP-2, PSD-95, and SYN in the hippocampus of CUMS model rats were assessed by western blotting. As shown in Figure 4, significant differences in the hippocampal protein levels of MAP-2, PSD-95 and SYN were found among the groups (F (3, 8) = 11.14, *P*=0.0032; F (3, 8) = 8.692, *P*=0.0067; and F (3, 8) = 9.509, *P*=0.0051). The protein expression levels of MAP-2, PSD-95, and SYN in the CUMS group were significantly lower than those in the control group (*P* < 0.05, *P* < 0.05, *P* < 0.05), whereas the treatments with EA and FLX increased the levels of these proteins (EA: *P* < 0.05, *P* < 0.05, and *P* < 0.05; FLX: *P* < 0.05, *P* < 0.05, and *P* < 0.05).

These results were confirmed by immunofluorescence staining, as shown in Figure 5. The relative fluorescence intensities of MAP-2, PSD-95, and SYN were significantly different (F (3, 8) = 12.02, *P*=0.0025; F (3, 8) = 12.81, *P*=0.0020; and F (3, 8) = 14.50, *P*=0.0013). Post hoc analyses showed that the relative fluorescence intensities of MAP-2, PSD-95, and SYN were lower in the CUMS group than in the control group (*P* < 0.05, *P* < 0.05, and *P* < 0.05), and EA treatment markedly increased the relative fluorescence intensities (*P* < 0.05, *P* < 0.05, and *P* < 0.05). FLX also reversed these changes (*P* < 0.05, *P* < 0.05, and *P* < 0.05), and the trend of these changes was generally consistent with the WB results.

### 3.3. EA Alleviated the Loss of Hippocampal Neurons

The morphology and number of hippocampal neurons in the CA3 region were observed by Nissl staining. As shown in Figures 6(a) and 6(b), significant differences in the numbers of positive neurons were found among the groups (F (3, 8) = 13.55, *P*=0.0017). Compared with the control group, the CUMS group exhibited obvious morphological changes (weak staining, a loose arrangement, and an irregular shape) and a significantly lower number of positive neurons (*P* < 0.05). Compared with the results obtained for the CUMS group, EA and FLX improved the histopathological features of the hippocampus and reversed the loss of Nissl bodies (EA: *P* < 0.05; FLX: *P* < 0.05).

### 3.4. EA Increased the Density of Dendritic Spines in the Hippocampus

The dendritic spine density in the CA3 region was then detected by Golgi staining (Figures 6(c) and 6(d)), which revealed significant differences among the groups (F (3, 12) = 45.22, *P* < 0.0001). Compared with that found in the control group, the density of dendritic spines in the CUMS group was significantly decreased (*P* < 0.05), and that found in CUMS rats treated with EA and FLX was significantly increased (*P* < 0.05, *P* < 0.05), which indicated that EA improved the density of dendritic spines in the hippocampus of CUMS model rats.

### 3.5. The GluN2B/CaMKII/CREB Signalling Pathway Was Involved in the EA Regulation of Depression-Like Behaviours and Neuronal Plasticity

To further explore the molecular mechanism through which EA exerts the abovementioned therapeutic effects, the protein levels of GluN2B, CaMKII, CREB, and p-CREB in the hippocampus were detected by western blotting. As shown in Figure 7, significant differences in the protein expression levels of GluN2B, CaMKII, and p-CREB were found among the groups (F (3, 8) = 7.411, *P*=0.0107; F (3, 8) = 7.169, *P*=0.0118; and F (3, 8) = 7.956, *P*=0.0087), but no differences in the levels of CREB were detected (F (3, 8) = 0.5843, *P*=0.6419). A post hoc analysis showed that the hippocampal protein levels of GluN2B and CaMKII in the CUMS group were significantly higher (*P* < 0.05 and *P* < 0.05) and that the level of p-CREB was significantly decreased (*P* < 0.05) compared with the levels found in the control group. In contrast, the EA group presented significantly lower hippocampal protein levels of GluN2B and CaMKII (*P* < 0.05 and *P* < 0.05) and significantly higher levels of p-CREB (*P* < 0.001) compared with those found in the CUMS group.

## 4. Discussion

In this study, we replicated a rat model of CUMS depression to observe the effects of EA on behaviour and synaptic plasticity and explore the possible underlying mechanisms. Our results suggest that 4 weeks of EA treatment can improve both CUMS-induced depression-like behaviour and hippocampal synaptic plasticity in rats, and the mechanism may be related to the inhibition of the GluN2B/CaMKII/CREB pathway.

As an important risk factor for mental illness, chronic stress is widely used as an animal model of mood disorders, and the CUMS model can simulate stress-induced depression [35], is widely used in preclinical research, and exhibits perfect aetiological, predictive, and face validity [36, 37]. Animal studies have shown that CUMS stress can cause behavioural symptoms of depression, such as an increased immobility time and reduced sucrose consumption [38, 39]. Consistently, our results showed that, after 28 days of CUMS induction, the rats exhibited significantly reduced sucrose consumption, significantly lower numbers of crossings, and significantly increased immobility times in the FST, whereas EA reversed these changes and exerted effects similar to those obtained with FLX. This finding shows that EA exerts a good antidepressant effect, which is consistent with some of our previous research results [33, 40].

Dendritic spines are the main sites of synapses between neurons, and the integrity of the dendritic spine structure and function is directly related to the regulation of learning, memory, and emotion [41]. Chronic stress leads to hippocampal structural remodelling and functional damage, including synaptic plasticity and dendritic atrophy [42]. Clinical studies have shown that the main causes of hippocampal atrophy in patients with severe depression are dendrite atrophy and spinous process reductions [43]. The helplessness and anhedonic behaviours of rodents have also been observed using an mTORC1 signal inhibitor (REDD1), which reduces the number of synapses [44]. In this study, the dendritic spine density was observed by Golgi staining. The results revealed significantly decreased densities in the CUMS group, which indicated that stress can decrease synaptic plasticity, and this finding is consistent with previously reported results [45, 46]. Notably, EA treatment significantly improved the dendritic spine density. Nissl bodies are a structural characteristic of the neuron cytoplasm, and their sensitivities change, as characterized by obvious dissolution or disappearance, upon the induction of neuronal damage by various factors. Therefore, Nissl staining is often used to evaluate the morphology and number of neurons. In this study, we observed the hippocampal CA3 regions and found that the model group exhibited irregularly shaped neurons and significantly reduced neuron numbers, which suggests that stress can cause neuronal damage. Both EA and positive drug administration significantly improved the number and structure of neurons.

Reductions in synaptic protein levels exert very harmful effects on synaptic function, and proteins such as MAP-2, SYN, and PSD-95 play important roles in the regulation of synaptic function [47]. MAP-2, a cytoskeletal protein that specifically exists in the dendritic branches of neurons, participates in the assembly of microtubules and stabilizes their growth [48, 49]. Located in the postsynaptic membrane, PSD-95 is an important indicator of the efficiency of information transmission between neurons and plays an important role in the stimulation and maintenance of synaptic structure and functional plasticity [50]. SYN is involved in the regulation of synaptic transmission efficiency and is the most abundant synaptic vesicle protein, and its distribution and density can indirectly reflect the number of synapses and the transmission efficiency [51]. Several studies have reported that chronic stress can decrease the expression of presynaptic and postsynaptic marker proteins, and antidepressant therapy can reverse these trends [17, 52, 53]. In this study, both western blotting and immunofluorescence revealed that the hippocampal protein levels of MAP-2, SYN, and PSD-95 were significantly reduced in the CUMS group and that EA upregulated their expression.

NMDAR, a heterologous complex comprised of the essential NR1 subunit and the regulatory GluN2 (GluN2A–D) subunit, plays an important role in regulating synaptic plasticity as well as learning and memory [24, 25]. However, NR2B is considered the most closely associated with depression [54]. It has been reported that GluN2A-containing NMDARs are mainly located in synapses and preferentially mediate cell survival. GluN2B-containing NMDARs mainly reside at extrasynaptic sites and are involved in cell death [55]. In adult mammals, GluN2B subunits are mainly expressed in the cortex and striatum, particularly in the hippocampus [56]. Animal studies have revealed that GluN2B protein expression is significantly upregulated in a rat model of depression [26]. In addition, patients who die from suicide exhibit a higher GluN2B mRNA level than patients who do not die from suicide [57]. Selective GluN2B antagonists also induce antidepressant responses in patients with treatment-resistant major depression [58]. Thus, inhibiting the excessive activation of GluN2B plays a key role in the treatment of depression [59].

Chronic stress can lead to the excessive accumulation of glutamate and to the overactivation of GluN2B-containing NMDARs [26], and these effects are followed by the opening of ion channels, which results in the influx of Ca^2+^ [60, 61]. CaMKII is an important molecule downstream of NMDAR, and its activity is mainly regulated by GluN2B-controlled calcium influx. The interaction between CaMKII and GluN2B plays an important role in the maintenance of synaptic strength and the induction of hippocampal central neuron dendrogenesis [62]. CaMKII activation further activates the downstream signal CREB, which regulates the phosphorylation of CREB and the expression of proteins related to synaptic plasticity [63–65]. Therefore, we speculate that EA improves the synaptic plasticity of depression models by inhibiting GluN2B activation and the downstream CaMKII/CREB pathway. We analysed the hippocampal protein levels of GluN2B, CaMKII, CREB, and p-CREB and found that CUMS significantly increased the levels of GluN2B and CaMKII, decreased those of p-CREB, and did not alter the protein levels of CREB. EA treatment reversed these changes, which suggests that the GluN2B/CaMKII/CREB signalling pathway is involved in the antidepressant effect and the improvement in synaptic plasticity obtained with EA.

In conclusion, this study found that EA can improve depression-like behaviour and synaptic plasticity in hippocampal neurons and that these effects are potentially related to the GluN2B/CaMKII/CREB signalling pathway. Our study suggests that EA is a promising therapeutic strategy for depression, but the precise mechanism needs further study.

## Figures and Tables

**Figure 1:** Experimental procedures.

**Figure 2:** Acupoint locations on the rat body where electroacupuncture was applied.

**Figure 3:** Effect of EA on depression-like behaviour. (a) Numbers of crossings in the OFT. (b) Number of rearings in the OFT. (c) Sucrose preference ratio in the SPT. (d) Immobility time in the FST. All the results are expressed as the means ± SEMs, *n* = 12 per group, ^*∗*^*P* < 0.05 compared with the control group, and ^#^*P* < 0.05 compared with the CUMS group.

**Figure 4:** Effect of EA on synaptic plasticity-related proteins. (a) Representative western blot bands of hippocampal MAP-2, PSD-95, and SYN. (b, c, d) Quantification of the relative hippocampal protein levels of MAP-2, PSD-95, and SYN. All results are expressed as the means ± SEMs, *n* = 3 per group, ^*∗*^*P* < 0.05 compared with the control group, and ^#^*P* < 0.05 compared with the CUMS group.

**Figure 5:** Immunofluorescence analysis of the effect of EA on synaptic plasticity-related proteins. (a, b, c) Representative images of MAP-2 (red), PSD-95 (red), and SYN (red) fluorescence staining in the hippocampal CA3 regions, nuclei stained with DAPI (blue). (d, e, f) The relative fluorescence intensities of MAP-2, PSD-95, and SYN in the hippocampal CA3 regions are semiquantitative. All results are expressed as the means ± SEMs, *n* = 3 per group, and scale bar = 50 *μ*m. ^*∗*^*P* < 0.05 compared with the control group; ^#^*P* < 0.05 compared with the CUMS group.

**Figure 6:** Nissl and Golgi staining in the hippocampus. (a) Representative images of Nissl staining in the hippocampal CA3 regions. Scale bar = 50 *μ*m. (b) Quantitative analysis of the neuron numbers in the hippocampal CA3 regions. (c) Representative images of dendritic spines in the hippocampal CA3 region of each group. Scale bar = 2.5 *μ*m. (d) Quantitative analysis of the dendritic spine density in the hippocampal CA3 region. All results are expressed as the means ± SEMs, *n* = 3 per group, ^*∗*^*P* < 0.05 compared with the control group, and ^#^*P* < 0.05 compared with the CUMS group.

**Figure 7:** Western blot analysis of the effect of EA on the GluN2B/CaMKII/CREB signalling pathway. (a) Representative western blot bands of hippocampal GluN2B, CaMKII, CREB, and p-CREB. (b–e) Quantification of the relative hippocampal protein levels of GluN2B, CaMKII, CREB, and p-CREB. All results are expressed as the means ± SEMs, *n* = 3 per group, ^*∗*^*P* < 0.05 compared with the control group, and ^#^*P* < 0.05 compared with the CUMS group.

## Data Availability

The figure data used to support the findings of this study are available from the first author upon request.
